# Isoquinoline Alkaloids and Indole Alkaloids Attenuate Aortic Atherosclerosis in Apolipoprotein E Deficient Mice: A Systematic Review and Meta-Analysis

**DOI:** 10.3389/fphar.2018.00602

**Published:** 2018-06-05

**Authors:** Yibing Zhang, Min Li, Xiangjun Li, Tong Zhang, Meng Qin, Liqun Ren

**Affiliations:** ^1^Department of Pharmacology and Toxicology, School of Pharmaceutical Sciences, Jilin University, Changchun, China; ^2^Department of Ophthalmology, First Hospital of Jilin University, Changchun, China

**Keywords:** meta-analysis, alkaloid, atherosclerosis, ApoE deficient mouse, natural compounds

## Abstract

**Background:** Several studies have attempted to relate the bioactive alkaloid with atherosclerotic cardiovascular diseases prevention in animal models, providing inconsistent results. Moreover, the direct anti-atherosclerotic effects of alkaloid have hardly been studied in patients. Therefore, the aim of this systematic review was to assess the reported effects of alkaloids on aortic atherosclerosis in ApoE^−/−^ mouse models.

**Methods**: Pubmed and Embase were searched to identify studies which estimated the effect of isolated alkaloids on atherosclerosis in apolipoprotein E deficient mice. Study quality was assessed using SYRCLE's risk of bias tool. We conducted a meta-analysis across 14 studies using a random-effect model to determine the overall effect of the alkaloids, and performed subgroup analyses to compare the effects of the isoquinolone alkaloids and indole alkaloids.

**Results:** The quality of the included studies was low in the majority of included studies. We clarified that alkaloid administration was significantly associated with reduced aortic atherosclerotic lesion area (SMD −3.19, 95% CI −3.88, −2.51). It is important to remark that the experimental characteristics of studies were quite diverse, and the methodological variability could also contribute to heterogeneity. Subgroup analyses suggested that the isoquinoline alkaloids (SMD −4.19, 95% CI −5.18, −3.20), and the indole alkaloids (SMD −2.73, 95% CI −3.56, −1.90) obviously decreased atherosclerotic burden.

**Conclusion:** Isoquinoline alkaloids and indole alkaloids appear to have a direct anti-atherosclerotic effect in ApoE^−/−^ mice. Besides the limitations of animal modal studies, this systematic review could provide an important reference for future preclinical animal trials of good quality and clinical development.

## Introduction

Atherosclerosis is one of the major causes for cardiovascular diseases including coronary heart disease (CHD), the leading cause of morbidity and mortality worldwide could be generally the cardiovascular disorders and CHD alone (Mozaffarian et al., 2016). Previous studies showed atherosclerosis was deeply linked with hypercholesterolemia via inflammation reactions (Cui et al., 2018). Despite the widespread use of statin-based lipid-lowering therapies, which has decreased CHD mortality rates, the global burden of this disease remains high. Identifying novel therapeutic strategies for more effective prevention and treatment in atherosclerosis, therefore, remains a topic of interest (Ford et al., 2018). So many researchers began to focus on new hopeful treatment of natural compounds, the compounds of natural origin have been shown to positively affect atherosclerosis, at least in experimental studies, for example, flavonoid, alkaloid, terpenoid, and many others (Chi et al., 2014; Pirillo and Catapano, 2015; Xiao et al., 2017; Ramanathan et al., 2018; Zhang et al., 2018).

Alkaloids are a group of naturally occurring chemical compounds that mostly contain basic nitrogen atoms. Alkaloids have a wide range of pharmacological activities, many have found use in traditional or modern medicine, or as starting points for drug discovery. Recently, alkaloid has received emerging interest from pharmacologists and health practitioners with its multi therapeutic effects, including hypocholesteremic capacity, anti-inflammatory, anti-oxidative, and anti-atherosclerotic properties (Jun et al., 2016). Extensive studies in animal models of hyperlipidaemia have also supported the beneficial effects of natural alkaloid to delay atherosclerotic progression. In addition, the most studied alkaloids are the isoquinolone alkaloids, the indole alkaloids, and purine alkaloids. Nevertheless, the relatively therapeutic effects of natural alkaloids have not been confirmed in patients.

Animal model is a valuable approach for preclinical research, which provides information for the treatment strategy of human diseases. ApoE deficient (ApoE^−/−^) mice can spontaneously develop atherosclerosis which covers the whole spectrum of human lesions. Indeed, they are known to develop a robust aortic atherosclerotic phenotype when fed a high-fat diet. In recent animal experiments of atherosclerosis, almost all the researches are carried out in ApoE deficient background. As a well-defined classical atherosclerotic model, substantial researches of anti-atherosclerotic administration have been performed in ApoE^−/−^ mice (Jawien, 2012; Tani et al., 2014; Sun et al., 2017). However, the general effect of alkaloids on atherosclerosis is still inconclusive, the effect of subgroup alkaloids is yet to be investigated, and the quality of the reported data should be appraised critically.

In order to comprehend the direct effects of alkaloids and to provide further information about the potential translation of the experimental results to humans, we therefore assessed the preventive effect of alkaloids on atherosclerosis in ApoE^−/−^ mice in this systematic review and meta-analysis.

## Materials and methods

### Review protocol

A protocol for this systematic review was prepared using SYRCLE's systematic review protocol format for animal intervention studies (https://www.syrcle.nl) (de Vries et al., 2015).

### Study identification

A systematic search (between January 2011 and February 2018) was conducted by comprehensive searches in two online databases (PubMed and EMBASE). The searches were designed and executed by an experience information specialist (ML). The search strategy consisted of two main components: atherosclerosis, and alkaloids, and results were limited to apolipoprotein E deficient mice. Key words included “atherosclerosis,” “atherogenesis,” “apolipoproteins e,” “apoe,” “mice,” and “alkaloids” as follows: (atherosclerosis OR atherogenesis) AND (“apolipoprotein^*^ e” OR apoe) AND (mice OR mouse) AND (alkaloids OR isoquinolone alkaloids OR indole alkaloids OR Berberine OR Caffeine). The reference lists of included studies and relevant reviews were hand searched to identify additional relevant studies. Searches were performed on February 12th 2018. Included studies were restricted to those published in English.

### Study selection

The selection procedure was performed by two independent reviewers (YZ and LR). References were exported to Endnote for removal of duplicates. Resulting titles and abstracts were screened for relevance. The following criteria were used for titles and abstract screening phase: (1) original research, defined as a study that presented original data and did not specifically state that it was a review; (2) study conducted in apoE deficient mice; (3) disease of interest (atherosclerosis); (4) intervention of interest (alkaloids). Subsequently, the full text manuscripts of eligible studies were reviewed. We finally included animal studies using ApoE^−/−^ mouse model, comparing alkaloid-treated animals with vehicle-treated controls, and reporting atherosclerotic lesion area as an outcome measure.

### Quality assessment of included studies

The SYRCLE's Risk of Bias tool was used to assess the risk of bias of all included studies (Hooijmans et al., 2014). Two independent investigators (YZ and XL) performed quality assessment of all included studies. Disagreements were resolved by discussion.

### Data extraction and study characteristics

Full text articles eligible for data extraction were independently assessed by three authors (YZ, ML, and LR) and results were later discussed in a consensus meeting. The data extracted included mouse age, sex and diet, alkaloid dose, duration and route of treatment, control and treatment group sample sizes, location of atherosclerosis area assessed, stain used for lesion assessment, and lesion area. Our outcome was the atherosclerotic lesion size measured as a percentage of the area or lesion area numerical value. Mean value, standard deviation (SD), and the number of animals per group were extracted. If relevant data were not available in the text but only presented in graphic form, obtaining the data by measuring the graphs using Adobe Photoshop 7.0.

### Data synthesis and statistical analysis

For the outcome measures of atherosclerotic lesion area, the standardized mean difference (SMD) was used as the effect measure. Data were expressed as standardized mean difference with 95% confidence intervals. If studies contained multiple independent groups (e.g., different alkaloid dose), they were treated as separate experiments. In five studies (Cai et al., 2013; Chen et al., 2014; Xu et al., 2014; Feng et al., 2017a; Zhu et al., 2018), the researchers used the same control group to compare multiple alkaloids or alkaloid doses. Consequently, the number of control animals was divided by the number of comparator groups to avoid a man-made expansion in sample size in the meta-analysis.

The use of multiple alkaloids, at different doses with different durations of treatment could lead to heterogeneity. We analyzed the data using a random effect model. I^2^ was used as a measure of heterogeneity. Heterogeneity above 30% was considered moderate, and heterogeneity above 50% was considered high. A meta-analysis was performed to evaluate the total effects of the administration of alkaloids on the outcome of atherosclerotic lesion area in ApoE^−/−^ mice. To explore potential causes of heterogeneity, predefined subgroup analyses were performed when subgroups contained data from at least three studies. Sub-analyses were conducted to investigate the general effect of isoquinoline alkaloids and indole alkaloids on atherosclerotic lesion area.

In addition, sensitivity analyses were conducted as to evaluate whether the findings were robust enough to the decisions made. Visual inspection of funnel plots was used to detect publication bias. Statistical analyses were performed using RevMan 5.3, and tests were considered significant when *P*-values were < 0.05.

## Results

### Study selection

The comprehensive search strategy on the effects of alkaloid on atherosclerosis in ApoE^−/−^ mouse models resulted in 632 records. References were exported to Endnote, after duplicates were removed, 567 studies were left. After title and abstract screening, 20 studies were screened full text for final inclusion. Four of these studies were excluded because atherosclerosis lesion area was not reported (Ching et al., 2013; Wang et al., 2015; Li et al., 2016; Yang et al., 2017), one study was excluded because a mixture of herbal medicines was administered (Ho et al., 2012), and one study was excluded for intervention combining with surgery (Son et al., 2012). At last, 14 eligible studies were included in this systematic review (Wang et al., 2011; Ching et al., 2012; Fujiwara et al., 2012; Mercer et al., 2012; Cai et al., 2013; Wei et al., 2013; Zhuang et al., 2013; Chen et al., 2014; Xu et al., 2014; Feng et al., 2017a,b; Jiang et al., 2017; Liu et al., 2017; Zhu et al., 2018), of which studies (total 21 animal experiments and 331 animals involved) could be embodied in the meta-analysis (Figure 1).

**Figure 1:** Flow diagram of the study identification and selection process.

### Study characteristics

The characteristics of the fourteen included studies are described in Table 1. The characteristics among these studies varied considerably. Only three studies used female animals, eight used male, and three studies didn't mention the gender of animals in their experiments. Mice received a normal-chow diet in five studies (Ching et al., 2012; Fujiwara et al., 2012; Mercer et al., 2012; Wei et al., 2013; Jiang et al., 2017); a high fat diet in nine studies containing either 21% fat and 1.25% cholesterol (Feng et al., 2017a,b), 42% fat and 0.2% cholesterol (Zhu et al., 2018), 32% fat and 1% cholesterol (Chen et al., 2014), 20% fat and 0.15% cholesterol (Xu et al., 2014), 16.6% fat, 10.6% sucrose and 1.3% cholesterol (Zhuang et al., 2013), the D12079B diet (Research Diets Inc,), containing 21% fat and 0.21% cholesterol (Wang et al., 2011), the D12108C diet (Research Diets Inc,), containing 20% fat and 1.25% cholesterol (Cai et al., 2013), and unmarked fat and cholesterol content (Liu et al., 2017). Administration timing and duration of alkaloids varied greatly. The age of the mice when alkaloid administration was initiated was 4 weeks in one study (Mercer et al., 2012), 5 weeks in two study (Wang et al., 2011; Zhu et al., 2018), 6 weeks in five studies (Fujiwara et al., 2012; Zhuang et al., 2013; Feng et al., 2017a,b; Liu et al., 2017), 8 weeks in three study (Cai et al., 2013; Xu et al., 2014; Jiang et al., 2017), 12 weeks in one study (Chen et al., 2014), and 16 weeks in two study (Ching et al., 2012; Wei et al., 2013). The duration of daily treatment varied between 4 weeks to 16 weeks. Besides, the characteristics of administration route differed substantially between the studies. Intragastric dosages between 10 and 150 mg/kg were most common, but intra-peritoneal, adding to the drinking water and chow administration was also used. Six studies administered the alkaloids via the intragastric route (Ching et al., 2012; Wei et al., 2013; Xu et al., 2014; Feng et al., 2017a,b; Jiang et al., 2017), three studies administered the alkaloids by adding it to the drinking water (Wang et al., 2011; Liu et al., 2017; Zhu et al., 2018), three studies administered the alkaloids by adding to the chow (Fujiwara et al., 2012; Mercer et al., 2012; Chen et al., 2014), and two studies administered the alkaloids via the intraperitoneal injection (Cai et al., 2013; Zhuang et al., 2013).

**Table 1:** Study characteristics of the included ApoE^−/−^ mouse model.

**Study**	**Alkaloid**	**Age**	**Gender**	**Diet**	**Study length**	**Dose**	**Route**	**Location of lesion area**	**Analysis**	**Staining**	**Groups and sample size**
Chen et al., 2014	Berberine dhBBR Di-MeBBR	12 w	Male	HFD	16 w	1 mg/kg/d 10 mg/kg/d 10 mg/kg/d	Chow	Aortic root to thoracic aorta	En face (longitudinal)	Oil red O	Model Control, n = 6 Berberine, n = 6 dhBBR, n = 6 Di-MeBBR, n = 6
Feng et al., 2017a	Coptisine	6 w	Male	HFD	12 w	150 mg/kg/d	IG	Aortic root	Cross sectional	Oil red O	Model Control, n = 6 Coptisine, n = 6
Feng et al., 2017b	Berberine 8-BBR-C16	6 w	Male	HFD	12 w	150 mg/kg/d	IG	Aortic sinus	Cross sectional	Oil red O	Model Control, n = 6 Berberine, n = 6 C16c, n = 6
Wang et al., 2011	Berberine	5 w	?	HFD	8 w	1 mmol/L	Drink	Aortic arch (ascending arch to 5 mm distal of left subclavian artery)	En face (longitudinal)	Sudan IV	Model Control, n = 7 Berberine, n = 7
Zhu et al., 2018	Berberine	5 w	Female	HFD	14 w	0.5 g/L	Drink	①Aortic root to iliac branches ②Aortic root	①En face (longitudinal) ②Cross sectional	①Oil red O ②HE	Model Control, n = 10;5 HFD-BBR, n = 10;5
Cai et al., 2013	Vinpocetine	8 w	Male	HFD	16 w	5 mg/kg/d	i.p.	①Aortic root to iliac branches ②Aortic root	①En face (longitudinal) ②Cross sectional	①Oil red O ②HE	Model Control, n = 7;7 Vinp, n = 7;7
Ching et al., 2012	Evodiamine	16w	Male	NCD	4w	10mg/kg/d	IG	Aortic root	Cross sectional	HE	Model Control, n = 10 Evo, n = 10
Wei et al., 2013	Evodiamine	16 w	Male	NCD	4 w	10 mg/kg/d	IG	Aortic sinus	Cross sectional	HE	Model Control, n = 12 Evo, n = 12
Xu et al., 2014	Rutaecarpine	8 w	Female	HFD	8 w	10 mg/kg/d 20 mg/kg/d 40 mg/kg/d	IG	Aortic root to iliac branches	En face (longitudinal)	Oil red O	Model Control, n = 12 RUT low, n = 12 RUT medium, n = 12 RUT high, n = 12
Zhuang et al., 2013	Vinpocetine	6 w	Male	HFD	12 w	5 mg/kg/d	i.p.	Aortic arch and thoracic aorta	En face (longitudinal)	Oil red O	Model Control, n = 5 Vinpocetine, n = 5
Fujiwara et al., 2012	Tomatidine	6 w	?	NCD	70 d	50 mg/kg/d	Chow	Aortic sinus	Cross sectional	Oil red O	Model Control, n = 10 Tomatidine, n = 10
Jiang et al., 2017	Leonurine	8 w	Male	NCD	8 w	10 mg/kg/d	IG	Aortic sinus	Cross sectional	Oil red O	Model Control, n = 15 Leonurine, n = 15
Liu et al., 2017	Caffeine	4 w	Female	NCD	12 w	0.05%	Chow	Aortic root to thoracic aorta	En face (longitudinal)	Nile red	Model Control, n = 10 Caffeine, n = 10
Mercer et al., 2012	Caffeine	6 w	?	HFD	14 w	400 μg/g	Drink	Aortic root	Cross sectional	HE	Model Control, n = 18 Caffeine, n = 15

*NCD, normal-chow diet; HFD, high-fat diet; Vinp, Vinpocetine; Evo, Evodiamine; RUT, rutaecarpine; IG, intragastric; i.p., intraperitoneal injection; HE, hematoxylin and eosin; ? = not mentioned*.

The 14 included studies collectively measured the effects of 11 unique alkaloids, at multiple doses in a total of 21 comparisons, based on the outcome of atherosclerotic lesion area. Seven studies measured cross sectional aortic lesion area in mice receiving alkaloids and controls (Ching et al., 2012; Fujiwara et al., 2012; Wei et al., 2013; Feng et al., 2017a,b; Jiang et al., 2017; Liu et al., 2017), all of the studies measured aortic lesion area at the level of the aortic root or sinus. Five studies measured En face (longitudinal) aortic lesion area (Wang et al., 2011; Mercer et al., 2012; Zhuang et al., 2013; Chen et al., 2014; Xu et al., 2014). Two studies measured both cross sectional and En face (longitudinal) aortic lesion area (Cai et al., 2013; Zhu et al., 2018). Of these, three study measured longitudinal aortic lesion area from the aortic root to the iliac branches (Cai et al., 2013; Xu et al., 2014; Zhu et al., 2018), three study measured longitudinal aortic lesion area from the aortic root to the thoracic aorta (Mercer et al., 2012; Zhuang et al., 2013; Chen et al., 2014), one study measured the aortic arch (ascending arch to 5 mm distal of left subclavian artery) (Wang et al., 2011).

### Risk of bias and quality of included studies

The results of the study quality and risk of bias assessment are shown in Figure 2. On account of this assessment, 4 (29%) of the studies declared that the allocation was randomized. For the background of animals was generally homogenous, most of the studies didn't mention the particular method of randomization. Moreover, the risk of bias due to random housing and random outcome assessment was unclear. Only one study (7%) mentioned that any blinding was applied during the experiment, but this was related to the outcome assessment. Besides, the risk of bias due to allocation concealment and blinded interventions was assessed as unclear or high risk. Eleven studies stated sufficient detail to assess that the groups were similar at baseline, the other three studies did not report all of the baseline characteristics we assessed. Only one study reported death rate of ApoE^−/−^ mice at the end of the experiment. In the other studies, the number of animals per group was either mentioned only once, resulting in an unclear risk of attrition bias. The risk of selective outcome reporting was unclear in all studies, since none of them reported whether the outcomes were pre-specified in a protocol, in addition, no study protocols were included with the publications. The risk of other biases was assessed as low: all of the authors declare that there are no conflicts of interest.

**Figure 2:** Risk of bias and quality assessment, score (%) per risk of bias item.

By using the risk of bias tool, we found out that reporting is poor and therefore the methodological quality of many studies is unclear. It shows that there is much room for improvement, since many items were shown “unclear” and only a few items were shown low risk only in very few studies.

### Analysis of the effects of alkaloid on atherosclerotic lesion area

We could include data of 21 comparisons from fourteen studies reported outcomes related to aortic atherosclerotic lesion area. As such, a total of 185 alkaloid administered and 146 vehicle control ApoE^−/−^ mice were included in the overall meta-analysis (Figure 3). The overall effect of the alkaloids was to significantly lower atherosclerotic lesion area compared with controls (SMD −3.19, 95%CI −3.88, −2.51). However, between- study heterogeneity was quite high (I^2^ = 70%). Sub-group analyses were conducted to compare the effects of the isoquinoline alkaloids and indole alkaloids on atherosclerotic lesion area. Administration of isoquinoline alkaloids, brought about a significant decrease in atherosclerotic lesion area (SMD −4.19, 95%CI −5.18, −3.20) in a total of 58 experimental mice (40 control mice were included) with lower heterogeneity (I^2^ = 16%). The indole alkaloids did obviously lower atherosclerotic lesion area (SMD −2.73, 95%CI −3.56, −1.90) with medium heterogeneity (I^2^ = 56%), based on data from a total of 77 experimental and 53 control mice (Figure 3). The other subclasses of alkaloids did not contain more than three studies, thus sub-group analyses was unable to be performed.

**Figure 3:** Forest plot of overall effect of alkaloids on atherosclerosis. Sub- analyses were conducted to assess the effect of isoquinoline alkaloids and indole alkaloids on atherosclerotic lesion area. SD, standard deviation; CI, confidence interval; Std, standard; IV, inverse variance; BBR, Berberine; Vinp, Vinpocetine; Evo, Evodiamine; RUT, rutaecarpine.

### Sensitivity analysis and publication bias

Sensitivity analysis by substituting fixed effect model for random effect model showed that the outcome of the meta-analysis did not change [SMD −3.19, (−3.88, −2.51) vs. −2.49, [−2.83, −2.16)]. The asymmetry in funnel plots indicated the presence of publication bias (Figure 4).

**Figure 4:** Funnel plot overseeing publication bias of included studies.

## Discussion

### Summary of main findings

The advantage of a preclinical model is to clearly determine atherosclerotic progression in response to a given intervention. Several animal experimental studies indicate that natural alkaloids have potential benefits for atherosclerosis. As an important bridge between basic medicine and clinical research, animal experimental studies are significant to test the safety and efficacy of the interventions and to determine whether new administrations can be applied to clinical trials (Anglemyer et al., 2015). Specifically, ApoE^−/−^ mouse is a well-established animal model for studying atherosclerosis. The principal characteristics and progression of atherosclerotic lesions in ApoE^−/−^ mice and human beings are evidently similar (Vasquez et al., 2012; Chen et al., 2015). This furthermore supported the reliable and applicable results from ApoE^−/−^ mouse models.

Classification by chemical structure is the most common method of alkaloids. The major classes of alkaloids which had been identified for their anti-atherosclerotic effects were isoquinoline alkaloids and indole alkaloids, included in five studies respectively. In sub-analyses limited to the alkaloid class, isoquinoline alkaloids and indole alkaloids significantly reduced atherosclerotic lesion area. Berberine and its derivatives were the most studied alkaloid in the included studies. Our current review is the first to systematically appraise the effect of alkaloids on atherosclerosis in ApoE^−/−^ mice, in order to provide scientific basis for clinical trials of cardiovascular diseases. The favorable efficacy results of the present meta-analysis are consistent with the findings of each individual study included in the review and confirm statistically the significant improvement in atherosclerosis treated with alkaloids.

### Heterogeneity

A large proportion of published animal studies have varying degrees of defects in their experimental designs, implementation, and reporting methods, which significantly affects the authenticity and reliability of these studies, and poses differences in replicating results (Bailoo et al., 2014; Lee et al., 2017). We found potential evidence of heterogeneity among our included studies, primarily in experimental diversity. As a possible explanation for the variety, heterogeneity was remarkable reduced after sub-group analyses in terms of the alkaloid chemical classification. In addition, the different starting age, the different duration of treatment, the different diet and gender could lead to diverse progress of the atherosclerosis and provoke different effect of interventions. ApoE^−/−^ mice feeding normal chow could spontaneously develop atherosclerotic lesions. Fatty streaks in the proximal aorta are found at 3 months of age (Flurkey et al., 2007). Indeed, lesions development is associated with age and males are more susceptible than females, and sturdy lesions do form on the high-fat diet as well (Liu et al., 2015).

Afterwards, in the present study the methodological diversity in the assessment of aortic atheroma resulted in a significant heterogeneity in analysis. The majority of studies measured cross sectional lesion area of the aortic root or sinus, the other studies measured En face (longitudinal) aortic lesion area, and two of studies evaluated atherosclerotic burden in both cross-sections and longitudinal-sections indeed.

### Limitations

We accept as limitation that although ApoE^−/−^ mouse models could help us comprehend the pathogenesis of atherosclerosis, the characteristics of atherosclerosis are somewhat different between ApoE^−/−^ mice and humans. Such as atherosclerotic plaque of humans always occur in the coronary artery, the carotid artery, and the iliac artery, yet the plaque tend to gather in the root of the aorta and the brachiocephalic artery in mice. That may cause by the difference of heart rate and hemodynamics between mice and of humans, which corresponds to a region that experiences turbulent blood flow. Moreover, the fact that those studies were performed in a life history phase from adolescence to mature adult comparing with humans (all studies chosen were earlier than the middle of lifespan) precludes their use as an adequate tool of modeling of atherosclerosis where age is a key factor, especially considering the age-dependent risk of atherosclerosis. Furthermore, in the included atherosclerotic studies, the interventions of alkaloid were almost started simultaneously at the beginning of experimentation, which were employed to evaluate their utility in the early treatment (prevention experiment), not the advanced treatment (treatment paradigm). Because atherosclerosis is often treated as an advanced disease in the clinic, it is important to seek more treatment studies affect pre-established atherosclerotic plaques.

There are some other limitations in this review. For instance, our present analysis demonstrated that the isoquinoline alkaloids and indole alkaloids could exert protective effects on atherosclerosis in apoE deficient mice. Studies of other small animal models, such as LDL receptor- deficient mice, rabbits, and hamsters were not included into this meta-analysis. The species-specific differences in lipoprotein metabolism and vascular physiology could limit the usefulness of these experimental atherosclerotic models (Zadelaar et al., 2007). In this sense, it is difficult to conclude the validity of the beneficial effect of alkaloid interventions in atheroma plaque in all those small laboratory models to human beings. Moreover, other alkaloids may also have a similar effect, which is yet to be explored. Lack of replicate studies assessing the same subclass alkaloid precluded the possibility of performing a subgroup-analysis by analyzing the effect of specific natural compounds such as caffeine, or tomatidine or leonurine in ApoE^−/−^ mice. However, beneficial properties of any laboratory atherosclerotic models should be demonstrated clearly by using evidence-based medicine.

Besides, the outcome of this current analysis was the effect of alkaloids on atherosclerosis. Efficacy was defined as a decrease in a measure of atherosclerotic lesion area. However, other parameters, such as lipid profiles and body weight, were not included in the study. During the administration process, alkaloids may have a lipid-lowering effect, which needs to be further studied. Of note, the sample size of previously performed experimentation is still relatively small. Hence, further animal investigations, including studies of atherosclerosis with larger sample sizes, would be beneficial in assessing the effects of alkaloids on atherosclerosis for human use.

### Clinical implications

Notwithstanding its limitation, this study does suggest that isoquinoline alkaloids and indole alkaloids have anti-atherosclerotic effects in cardiovascular diseases and reduce atherosclerotic cardiovascular risk. Animal research data can generate and verify meaningful clinical hypotheses, reducing the potential risk to human trials. Hence, studies of human disease are often developed and improved upon as the result of animal experimentation. Globally speaking, large scale, prospective, and well-designed animal studies should be needed to deepen our knowledge concerning the causative role of alkaloid in atherosclerosis in the future.

## Conclusion

The alkaloids treatment performed on ApoE^−/−^ mice reported consistent findings that were confirmed by the present meta-analysis. Based on the coherent results, isoquinoline alkaloids, and indole alkaloids could potentially have a therapeutic effect on atherosclerosis. This analysis also reinforces the need for adequate standardization of atherosclerosis studies in preclinical models, and the pharmacological therapeutic effect of alkaloid merits future clinical studies. More human RCTs are needed before a conclusion regarding the anti-atherosclerotic effects of alkaloids in patients can be reached.

## Author contributions

LR designed the study and reviewed the draft. YZ conducted the analyses and writed the original draft. ML completed the methodology of study. XL performed the data curation. TZ collected the data. MQ done the work of statistics.

### Conflict of interest statement

The authors declare that the research was conducted in the absence of any commercial or financial relationships that could be construed as a potential conflict of interest.
